# Effects of Changyu Daotan Decoction on Depression via Restoration of Mice Hippocampus and Alteration of Expression of Relevant Neurotrophic Factors

**DOI:** 10.1155/2022/5750647

**Published:** 2022-08-29

**Authors:** Suifeng Zhang, Qian Chen, Lirong Wu, Ke Sun, Xiaofang Lan, Xin Xie, Junfeng Yan

**Affiliations:** ^1^Department of Spleen and Stomach Diseases, Chongqing Traditional Chinese Medicine Hospital, Chongqing, China; ^2^Department of Encephalopathy, Chongqing Traditional Chinese Medicine Hospital, Chongqing, China

## Abstract

Depression, a sort of common psychological disorder, is a serious hazard to people's health and social progress. Conventional clinical means for this disorder nowadays are mostly chemical medicine treatments accompanied by psychological counseling. Chinese application of using TCM to treat mental diseases like depression could be traced from hundreds of years ago, in comparison to the long-term depression course and the chemical medicine administration demerits like side effects and resistance, traditional Chinese medicines are milder, more lasting, stable and are the optimal choice for perennial depression treatment. This study was committed to making a comprehensive investigation of Changyu Daotan Decoction's efficacy in the depression mice model, and it turned out that the Changyu Daotan Decoction was capable of restoring the hippocampus of the depression mice and altering the expressions of neurotrophic factors (the expressions of *β*-Catenin, cyclin D1 and in GSK-3*β* BDNF, GFAP, NGF, and Wnt signaling pathways). Results of metabonomics analysis showed that the contents of GABA, His, Tyr, Trp, PA, and 5-HIAA in the mice of the Changyu Daotan Decoction group were restored after administration and showed a conspicuous relevance with the metabolic.

## 1. Introduction

Depression, a highly prevalent and recrudescent mental disorder, is clinically featured with black mood, anhedonia, and slow thinking. Patients with severe depression are prone to committing suicide, and it was reported that the prevalence of depression has been increasing year by year [1–3]. Up to now, there are at least about 350 million people suffering from depression, and this horde is likely to grow to be the first in the global disease burden in 2030 [4, 5]. However, the pathogenesis of depression is too complicated to be figured out, perhaps related to those factors such as genetics, immunology, psychology, and social environment [6].

The synaptic plasticity is inclusive of neurogenesis, axon branching, dendrite, and synaptogenesis; and current evidence suggests that some impairments of this aspect might happen in certain brain regions like the hippocampus and these lesions are in close association with an abnormal expression of neurotrophic factors, which are assumed to be the very factor of depression pathophysiology [7]. Based on the fact that the regeneration capacity of damaged hippocampal nerves is highly correlated with the onset and development of depression, many antidepressants treat depression by enhancing the regeneration capacity of hippocampal nerves [8].

Metabolomics, a newly emerging discipline, is a research method reliant on systems biology. Its principle is to guide the exploration of the relationship between metabolites and physiological and pathological changes and the mechanism of drug therapy by analyzing endogenous small molecule metabolites and their associated metabolic pathways. Metabolomics has been widely introduced in various aspects of the medical field, inclusive of disease diagnosis, pharmacological toxicology, new drug development, drug screening, etc. In recent years, this method has been applied more and more in the study on depression, which will help to elucidate its pathogenesis and development of antidepressant drugs.

This study worked to investigate the therapeutic effect of Changyu Daotan Decoction on mice with depression, so as to figure out valuable information and insights for associated research on depression.

## 2. Materials and Methods

### 2.1. The Animals

Forty SPF ICR mice were placed in the animal house and treated with the adaptive feeding of day and night alternately from 12 h to 12 h for 7 d. The experimental animals were given free access to drink and eat. Afterward, all the mice were randomly split up into different groups (blank group, model group, Changyu Daotan Decoction group, and positive control group) (10 mice in each group).

### 2.2. Changyu Daotan Decoction

Changyu Daotan Decoction, prescription: Shichangpu 15 g, Guangyujin 15 g, Polygala 15 g, Fried Shanzhi 10 g, Fandanpi 10 g, French Pinellia 15 g, Chi Fuling 15 g, Dannanxing 10 g, *Citrus aurantium* 10 g, 10 g of fine wood. Decoction in water, 1 dose per day, 2 times in the morning and evening, 4 weeks as a course of treatment.

### 2.3. Establishment of Animal Model

A revamped P.Willner model of chronic unforeseeable sexual stimulation was exploited to establish the model of the depression mice of other groups except the blank group. These treatments included ice water swimming (4°C, 5 min), heat stress (45°C, 5 min), fasting and water prohibition (24 h), tail clamping (hemostatic forceps were used to clamp 1 cm away from the tail tip of the mouse for 1 min), restriction and restriction of movement (1 h), wet padding and tilting the cage (24 h), and day and night reversal (indoor light as the principle). One of these treatments was randomly imposed and each treatment was used an average of 3 times per day. The same treatment of stimulus was not repeated in the same individuals over two days, and the modeling was lasted for a total of 21 days.

### 2.4. Behavioral Test Analysis

After modeling, mice were subjected to behavioral tests including sucrose water preference trial and a forced swimming trial.

#### 2.4.1. Sucrose preference test

Mice were first fed with sucralose water adaptively for 2 days for a total of 48 hours (during the adaptation process, it was noted that the position of sucralose water bottle was changed with that of the ordinary water bottle for 12 hours to avoid position preference in mice). The weight of residual sucrose and normal water after feeding was measured once daily. After the adaptation treatment (48 h later), all groups were treated with water fasting for 12 hours, and then the supply of sucrose water, ordinary water, and food was successively restored. After 12 h, the residual weight of sucrose water and ordinary water was determined, and the experimental results of sucrose water were recorded.

#### 2.4.2. Tail suspension experiment

The 1/3 of the mouse rear tail was fixed with adhesive tape, suspended on the scaffold, and the mouse head was kept 15 cm away from the table, and the subsequent behavior of the mouse was recorded by the camera. The camera background showed obvious contrast with mouse fur color, and C57 mice used white background. The timing was stopped after 5 min, and SuperTst software was used for recording.

#### 2.4.3. Forced swimming

This experimental method is a behavioral desperation experiment, which simulates an unavoidable oppressive environment by placing an animal in a confined environment (such as water) in which it desperately tries to escape but cannot. After a period of time, the animals show a typical immobile state. A series of parameters in the process of hopeless immobile state in experimental animals were observed and recorded, which can be used to evaluate the effect of antidepressant and depressant. The mice were put into a transparent plexigrate glass tank with a diameter of 10 cm and a height of 25 cm, with a depth of 15 cm and a water temperature of 25. The total immobility time of the mice for 5 min was recorded, which reflected the helplessness of the animals. The related parameters were recorded by SuperFst software.

### 2.5. Treating

After the modeling was established, Changyu Daotan Decoction group was given Changyu Daotan Decoction (3.9 g/kg) by gavage. Accordingly, the positive control group was given Sertraline Hydrochloride Tablets (SHT) (0.83 mg, kg) by intragastric administration. The Blank group and model group were given the same amount of normal saline.

### 2.6. Sampling

The experiment ended 3 weeks after administration. Mice were given with an intraperitoneal injection of pentobarbital sodium (50 mg/kg) to anesthetize, which were then sacrificed with the neck dislocation method. Part of mice's hippocampus tissues was quick-frozen with liquid nitrogen and kept in −80°C refrigerator for further usage, and another part of the tissues was homogenized and stored in −80°C refrigerator, and the rest were fixed with 4% neutral formaldehyde. The purpose of collecting mouse hippocampus tissue was used for Western Blot, Nissl staining, and immunohistochemistry to determine the structural changes of hippocampal tissue and the expression changes of related neural factors.

### 2.7. Western Blot

An appropriate amount of mouse hippocampal tissue was taken, and 1 mL of cell lysate was added into it. The mixture was fully ground and lysed on ice for 1 h, then centrifugated at 12 000 g for 20 min. The mixture was supernatant with 5X SDS-loading Buffer added and boiled at 100°C for 10 min before centrifugation. The samples were first treated with SDS-PAGE electrophoresis method and then transferred onto PVDF membrane. PVDF membrane was sealed with 5% defatted milk powder at room temperature for 1 h, and then incubated with the primary antibodies (1 : 1000 dilution) of *β*-catenin (ABclonal, A19657), GSK3*β* (ABclonal, A11731), cyclin D1 (Abclonal, A19038) and *β*-actin (ABclonal, AC026); afterward, the mixture was incubated overnight at 4°C. The treated PVDF membrane was washed with TBST for 5 min, repeated 3 times. The PVDF membrane was then placed in a blocking solution diluted secondary antibody (1 : 2000, ABclonal, AS014) and incubated at room temperature for 1 h. These PVDF membranes were washed with TBST for 5 min, repeated 3 times, then ECL chemiluminescence solution was dropped onto the membranes and X-ray development was performed in a darkroom.

### 2.8. Nissl's Staining

Fresh Seahorse central area tissue was taken and fixed in 10% neutral formalin solution for 24 h, and subsequently subjected to conventional dehydration, embedding, sectioning, and dewaxing. The 5 *μ*m thick slices were immersed in Cresyl Violet dye and soaked at 56°C for 1 h, after which the excess dye was rinsed with deionized water. The sections were treated with Nissl Differentiation for several seconds to 2 min (under the microscope until the background is nearly colorless). The slices were rapidly dehydrated with anhydrous ethanol, made transparent with xylene, and sealed with neutral resin. The slice images were collected and accomplished on the platform of the Mshot MF53 microscope produced by Guangzhou Mingmei Optoelectronic Technology Co., LTD.

### 2.9. Immunohistochemistry

After the operations of conventional dehydration, embedding, slicing, and dewaxing, the 5 *μ*m thick slices were treated with 3% hydrogen peroxide at room temperature for 15 min. The specimens were cleaned 3 times with PBS, 5 min each time. The sample was then sealed in goat serum at room temperature for 30 min, after which it was removed and the sealing solution was shaken dry (without rinsing). The samples were then incubated with primary antibody at 4°C (dilution ratio: 1 : 500) overnight and washed with PBS for 3 times for 5 min each time. The samples were placed in the secondary antibody (HRP labeled) working solution and incubated at room temperature for 1.5 h, then washed with PBS for 3 times, 5 min each time. The samples were placed in DAB for chromogenic treatment for 10 min (avoid the light), then washed twice with distilled water for 5 min each time, and redyed with hematoxylin for 5 min. Those samples were rinsed with tap water until they turned blue and then treated with 1% HCL ethanol for 5s. Finally, the samples were dehydrated by placing them in 95% ethanol for 2 min and then replaced with new 95% ethanol for another 2 min. These samples were then transparented with xylene for 5 min, followed by fresh xylene for another 5 min; after that, the samples were sealed with neutral resin. The section was observed and the image was collected by Mshot MF53 inverted microscope produced by Guangzhou Mingmei Optoelectronic Technology Co., LTD. The nucleus appeared blue under the microscope. Antibodies used: HRP-labeled goat anti-rabbit IgG (*H* + *L*) (1 : 50, Biyuntian, A0208), HRP Goat Anti-Mouse IgG (*H* + *L*) (1 : 200, ABclonal, AS003), BDNF Mouse mAb (1 : 200, ABclonal, A18129), GFAP Rabbit mAb (1 : 200, ABclonal, A19058), Nestin Rabbit pAb (1 : 200, ABclonal, A11861), NGF Rabbit pAb (1 : 200, ABclonal, A14216), and *β*-Tubulin Rabbit pAb (1 : 200, ABclonal, AC008).

### 2.10. UHPLC-MS Detection

The vacuum-dried solids were redissolved with 100 *μ*L 50% methanol. The solution was centrifuged at 4°C at 12000 g, and the supernatant was transferred to the injection bottle. The separation was carried out on a BEHC18 column (2.1 mm × 100 mm, 1.7 *μ*m) ultra-performance liquid chromatography platform. The injection volume in this experiment was 5 *μ*L. Mobile phase A: 0.1% formic acid-acetonitrile; mobile phase B: 0.1% formic acid - water. The flow rate was 0.35 mL/min, and the column temperature was 40°C. The chromatographic gradient was 0–0.5 min, 1% A; 0.5–3.5 min, 1–53% A; 3.5–7.5 min, 53–70%a; 7.5–9 min, 70–90%a; 9–13 min, 90% A; 13.1–15 min, and the gradient returns 1% A. In order to ensure the stability of the analysis system, quality control sample analysis is used at the beginning and end of each analysis. Positive and negative ion mode ESI source was used for mass spectrometry data collection. Specific scanning parameters were as follows: capillary voltage 4 kV for positive ion mode, 3.5 kV for negative ion mode; atomization temperature 330°C; atomizing gas flow rate of 10 L/min; fragmentation voltage 100 V; screening voltage 65 V; scanning range M/*Z* 70–1100; the scanning speed was 1.5 spectra/SEC [9, 10].

### 2.11. Metabolite Extraction

Accurately weigh an appropriate amount of brain tissue samples from the model group and drug treatment group into 2 mL EP tubes, add 600 *μ*L of 10% formic acid methanol solution-H2O (1 : 1.V/V) solution, add 2 steel balls, and vortex for 30 s; put it into a tissue grinder 55 Hz for 60 s, repeated twice; centrifuge at 12,000 rpm for 5 min at 4°C, take 100 *μ*L of the supernatant, accurately add 100 *μ*L of the isotope internal standard with a concentration of 100 ppb, vortex for 30 s, and the supernatant exceeds 0.22 filter with *μ*m membrane, add the filtrate into the detection bottle, and use it as a low-concentration substance detection sample; take 10 *μ*L of the original supernatant, add 490 *μ*L of 10% formic acid methanol-H2O (1 : 1.V/V) solution, and vortex for 30 s, take 100 *μ*L of the diluted sample, add 100 *μ*L of the isotope internal standard with a concentration of 100 ppb, vortex for 30 s, filter the supernatant through a 0.22 *μ*m membrane, and add the filtrate to the detection bottle as a high-concentration substance detection sample.

### 2.12. Bioinformatic Analysis

LC-MS data preprocessing is inclusive of peak matching, retention time correction, variable integration, data standardization, and other steps, and this course is mainly completed on the *R* platform loaded with the XCMS toolkit. In this section, the bandwidth was set to 15 sec, peak spread was 5–30 sec, and other parameters were default. The preprocessed data were imported into EZinfo in a matrix form to realize principal component analysis (PCA) and orthogonal partial least squares discriminant analysis (OPLS-DA). Hierarchical Clustering Analysis (HCA) was produced with imported MetaboAnalyst. Kruskal–Wallis test, Student's *t*-test, and logistic regression analysis were enforced on *R* platform to evaluate the influence of confounding factors [11, 12].

### 2.13. Statistical Analysis

The data analysis in this experiment was assisted and accomplished with Graph Pad Prism 7.0 software. Comparison between multiple groups in the experimental data was realized by one-way ANOVA, and comparison between groups was implemented with *t*-test. Parameter with *P* < 0.05 was statistically different.

## 3. Results

### 3.1. Changyu Daotan Decoction Offset the Depressive and Anxiety-like Symptoms of Mice

After sucrose water preference trial, tail suspension trial, and forced swimming, mice showed the decline in sucrose water preference rate (Figure 1(a)), and the increasing time span in both forced swimming (Figure 1(b)) and suspended tail immovability (Figure 1(c)). Subsequent behavioral tests showed that the model mice manifested declining responds in both autonomic and exploratory behaviors and tension, and worse behavioral helplessness and anhedonia under a novel environment, which indicated that the depressed mouse model was successfully replicated. After treatment with Changyu Daotan Decoction and sertraline hydrochloride tablets, the proportion of mice partial to sucrose water was escalated in strong contrast to the control group (*P* < 0.05), while the forced swimming and tail suspension immobility time of mice was dropped.

Through observation, it was found that the hippocampal neurons of mice in the control group were arranged neatly with intact structure, where the purplish blue Nissl bodies were abundant to be seen; on the contrary, the structure of neurons in the mice of the model group was disorganized with their number conspicuously decreased, where a large number of Nissl bodies were disappeared. In addition, the neuron structure in the mice of Changyu Daotan Decoction group was only slightly impaired, where the number of Nissl bodies turned increased; furthermore, the number of neurons and Nissl bodies in the mice of the positive control group were increased in a notable contrast to the Changyu Daotan Decoction group (Figure 1(d)).

BDNF is a very important cerebral neurotrophic factor, a wide range protector to neuro and regenerative function accelerator [13], and is a crucial marker protein in both the pathogenesis and the treatment of depression [14]. Reducing expression of BDNF in depression mice was increased after the treatment of Changyu Daotan Decoction, whose content was nearly up to that of the positive control. Alteration in GFAP content is pertinent to the onset and the development of neurological disease [14], and one of the pathophysiological mechanisms of major depression is the decrease and dysfunction of astrocytes [15]. In this experiment, the GFAP expression in the model group was conspicuously decreased; by comparison, the expression level of GFAP in Changyu Daotan Decoction group increased in both the positive control group and Changyu Daotan Decoction group. These findings were fitted with the evidence above.

NESTIN is a specific marker of neural stem cells, which is highly expressed in the nerve cells of patients with depression. A targeting treatment is able to reduce the expression level of NESTIN. Decreasing NGF expression in brain tissue would lead to morphological damage and affect the function of neurons in the hippocampus and cortex, and then eventually result in the occurrence of depression [16]. Our results revealed that the expression of NGF in depression mice turned greatly lower when compared with the control group. After Changyu Daotan Decoction treatment, expression of NGF in depression mice was similar to the positive control, both of which were increased significantly in comparison to the control group. On the other head, by comparison with the control group, expression of Tuj-1 in the model group was lessened, while that in Changyu Daotan Decoction group and positive control group were increased (Figure 2).

### 3.2. Effect of Changyu Daotan Decoction on Depression Mice through Wnt Signaling Pathway

Prior studies have demonstrated that GSK-3*β* is a key therapeutic target for mood disorders, and interference in GSK-3*β* activity is necessary for the rapid effect of ketamine antidepressants [17–20]. *β* -Catenin is also a neuropsychiatric-disorder molecule, participant in depression, and mediates resilience to stress [21–23] Cyclin D1 is highly correlated with cellular proliferation and differentiation and it is also an important target gene in the Wnt signaling pathway. Pertinent studies have found that high levels of Cyclin D1 and C-myc are in close association with *β*-catenin accumulation and the impairment of Wnt signaling pathway out of mutation [24]. Compared with the control group, the protein levels of *β*-catenin and cyclin D1 were signally decreased in the model mice of depression, while expression of GSK3*β* was significantly increased. After administration, we found both the expressions of *β*-catenin and cyclin D1 increased in Changyu Daotan Decoction and positive group, while the expression of GSK3*β* decreased (Figure 3).

Multivariate statistical analysis PCA analysis showed that the Blank control group and Changyu Daotan Decoction group shared a tendency to separate and clustered into two groups, which was effectively differentiated, with R2X values of 0.862, 0.868, 0.862, 0.88, 0.919, and 0.851, respectively, indicating significant differences among each group (Figure 4). In the dispersion point diagram of OPLS-DA model (Figure 5), the separation of the normal group and model group was obvious. In Figure 5(a)–5(f), R2X were 0.986, 0.964, 0.935, 0.957, 0.948, and 0.955, respectively. R2Y were 0.989, 0.997, 0.951, 0.977, 0.999, and 0.995, respectively. Q2 was 0.391, −0.355, 0.698, 0.165, 0.78, 0.873, respectively. Then, a substitution test was conducted on the model, and the results were shown in Figure 6. The intercept of Q2 in each group on the *Y*-axis was all less than 0, indicating that the model was not over-fitted, and differential metabolites could be screened accordingly.

### 3.3. Differences in Metabolites amid Samples

Metabolomics analysis showed that there were differences amid the metabolites in different groups. Versus the control group, the RNA levels of GABA, Gln, His, Tyr, Trp, PA, 5-HIAA, and Kyn in model group were increased, while the contents of their proteins were decreased after treatment with Changyu Daotan Decoction (Figure 7). *Z*-score (standard score) is a parameter to measure the level of metabolite content at the same level, and there were differences in metabolite content at the same level within different groups (Figure 8). Metabolite correlation revealed that the alterations of metabolites in each group were synergistic (Figure 9). Compared with the control group, GABA was positively correlated with Gln, His, Tyr, Trp, PA, *E*, 5-HIAA, and Kyn; expressions of His, Tyr, PA, *E*, and Kyn stood a positive correlation with Gln expression; expressions of Tyr, Trp, *E*, and 5-HIAA stood a positive correlation with the His. Besides, there was a positive correlation in the comparison of Changyu Daotan Decoction group and model group that expressions of Gln, His, Tyr, Trp, PA, *E*, 5-HIAA, Kyn versus the GABA; expression of Glu was negatively correlated with the GABA, His, Tyr, Trp, PA, *E,* and 5-HIAA; the His, Tyr, and Kyn were positively correlated with the Gln. On the basis of the information provided by the KEGG database, we plotted the possible upstream-downstream relationships amid the detected metabolites on a graph (Figure 10).

## 4. Discussion

Depression is a category of emotion disorders, whose main clinical manifestations are remarkable and long-lasting mood depression, thinking retardation, cognitive impairment, will activity decline and physical symptoms [25]. Medicine treatment is the mainstream means for depression [26]. Conventional single-target antidepressants are not effective in depression treatment, while traditional Chinese medicine has long been utilized to treat mental diseases [27]. In this study, the preference of mice in model group to sucrose water was decreased in a significant contrast to control group, while the forced swimming and tail suspension immobility time turned increased; when compared with model group, the mice in Changyu Daotan Decoction group showed a significant increase in their preference to sucrose water, suggesting that Changyu Daotan Decoction has a certain therapeutic effect on depression mice.

The hippocampus is an indispensable player in orchestrating stress responses and it is also in charge of learning, memory and associated with mood disorders; studies have found that the hippocampus is sometimes susceptible to psychological impairments [28]. It was found that the structure of hippocampal neurons in depressed mice was disordered and the number of neurons was decreased significantly, where Nissl bodies were greatly disappeared.

BDNF is a member of the neurotrophic factor family, a protein highly expressed in the hippocampus and prefrontal cortex. The BDNF protein is implicated in the pathogenesis of depression, and is also relevant to cell plasticity, cell cascade death, and the cell survival proteins about neuronal proliferation and maintenance [29]. Thus, mouse cases of depression showed a down-regulated BDNF expression in the hippocampus. GFAP levels reflect changes in astrocytes, which is a protein that promotes the secretion of inflammatory mediators. Over-expression of GFAP leads to hippocampal nerve damage and subsequent cognitive impairment [30]. Endogenous neural stem cells (NSCS) are multipotent stem cells that would be differentiated into neurons and glial cells under certain conditions. Nestin is a specific marker of neural stem cells [31, 32]. It has been demonstrated that depressive-like behavior in animals with neuronal damage and traumatic brain injury can lead to increased Nestin expression [33, 34]. In contrast, the proliferation of neural stem cells in the hippocampal region was significantly increased after depression treatment [35]. The expression of Nestin did not change significantly in several groups. Decreasing expression of NGF in brain tissue brings about the morphological damage of neurons in hippocampus and cortex, producing impairment to neuron function and resulting in the onset of depression [16]. Neuron damage and synaptic differentiation disorder beget down-regulation of Tuj-1; in that context, Tuj-1 is deemed as a specific marker of synaptic differentiation [36]. This study proves that Changyu Daotan Decoction can increase BDNF, NGF, Tuj-1, and GFAP, it is speculated that it protects hippocampal neurons by promoting further proliferation and differentiation of Nestin into astrocytes. After the neurons reach the normal level, that is, the neural stem cells are gradually replaced by astrocytes and stop their expression, and the neural stem cells reach the normal level, thus playing the role of protecting the hippocampal neurons.

Glycogen synthase kinase-3*β* (GSK-3*β*) is a constitutively active molecule under basic conditions, an ubiquitous serine/threonine protein kinase. Specific GSK-3*β* inhibitors are endowed with antidepressant effects, and they are able to alleviate the depression-like behavior in those animal models with depression [37]. *β*-catenin is a substrate for GSK-3*β*, whose expression in the hippocampus is deemed as a bio-marker of antidepressant behavior in clinical practice [38, 39]. Cyclin D1 is an important cyclin protein regulating cellular proliferation and differentiation, and it is also a critical target gene in the Wnt signaling pathway. Previous studies showed that overexpression of Cyclin D1 is in a close relation to *β* -catenin accumulation and the defective mutations in the Wnt signaling pathway [24]. Our study showed that Changyu Daotan Decoction produces an alteration in the GSK-3*β*, *β*-catenin, and Cyclin D1 expressions in the mouse hippocampus, alleviating mouse depressive symptoms in a way of mediating Wnt signaling pathway.

The pathogenesis of depression is closely related to central neurotransmitters [40]. There is increasing evidence that depression is caused by hypothalamic-pituitary-adrenal axis dysfunction, decreased neurotransmitter secretion, neuroinflammation, oxidative nitrosation stress, decreased cellular proliferation, aberrant cytokine secretion, diminishing neurotrophic factor levels, and neuroplasticity disorders [41, 42]. GABA is a cerebral inhibitory neurotransmitter system in charge of the overall control and regulating fine-tuning of excitatory transmission, whose function would be disrupted by stress and depression [43]. Metabonomic data of this experiment showed that GABA, His, Tyr, Trp, PA, and 5-HIAA contents were increased in the model group, the contents of which in depression mice were inhibited through Changyu Daotan Decoction treatment. We also found a correlation between metabolites: Gln, His, Tyr, Trp, PA, *E*, 5-HIAA, and Kyn expression in Changyu Daotan Decoction and model group showed a positive correlation with GABA content. As part of glial cell-neuron communication, Gln-Glu-GABA cycle is a considerable sector in excitatory and inhibitory neurotransmission [44]. Metabolic pathway analysis revealed interactions between Gln, Glu, and GABA, which can be interconverted through different intermediates. This reminds us that metabolites are interconvertible and that multiple metabolites play an important role in the treatment of depression. The results will provide ideas for the treatment of depression, such as how we can alter the levels of metabolites through medication or diet to facilitate the recovery of depressed patients.

## 5. Conclusion

In this study, Changyu Daotan Decoction was used to treat depression model mice, and the changes in hippocampal tissue structure and neurotrophic factor expression were measured. In addition, Changyu Daotan Decoction could alter the expressions of GSK-3*β*, *β*-catenin, and cyclin D1 in the hippocampus of mice. Metabolomics showed that Changyu Daotan Decoction could improve the content of neurotransmitters in depression model mice. This study shows that Changyu Daotan Decoction may have a therapeutic effect on depressed patients, but this is also the shortcoming of this paper, that is, it has not been validated clinically.

## Figures and Tables

**Figure 1:** (a) Sucrose water preference trial, (b) tail suspension trial, and (c) forced swimming trial were to verify the modeling establishment, (d) Nissl's staining was performed to observe the hippocampal structure. CDD: Changyu Daotan Decoction group; SHT: positive control group; with control group as the reference, ^*∗*^*P* < 0.05, ^*∗∗*^*P* < 0.01, ^*∗∗∗*^*P* < 0.001; with model group as the reference, ^#^*P* < 0.05, ^##^*P* < 0.01, ^###^*P* < 0.001.

**Figure 2:** Immunohistochemistry detection on the expression of BDNF, GFAP, NESTIN, NGF, and Tuj-1 proteins. CDD: Changyu Daotan Decoction group; SHT: positive control group; ^*∗*^: Compared to Control group,^*∗*^*P* < 0.05, ^*∗∗*^*P* < 0.01, ^*∗∗∗*^*P* < 0.001. ^#^: Compared to Model group, ^#^*P* < 0.05, ^##^*P* < 0.01, ^###^*P* < 0.001.

**Figure 3:** (a) Western blot detection on *β*-catenin, GSK3*β*, and Cyclin D1 expressions. (b) Analysis on *β*-catenin relative expression. (c) Analysis on the relative expression of GSK3*β*. (d) Analysis of cyclin D1 relative expression. CDD: Changyu Daotan Decoction; SHT: positive control group; with the control group as the reference, ^*∗∗∗*^*P* < 0.001.

**Figure 4:** Analysis of main components. (a) Blank and model groups; (b) Blank group and Changyu Daotan Decoction group; (c) Model group and Changyu Daotan Decoction group; (d) Blank group and positive control group; (e) Model group and positive control group; (f) Changyu Daotan Decoction group and positive control group. A stands for the blank group; B represents model group, C represents Changyu Daotan Decoction group, and C represents positive control group.

**Figure 5:** OPLS-DA model scores scatter diagram. (a) Blank and model groups; (b) Blank group and Changyu Daotan Decoction group; (c) Model group and Changyu Daotan Decoction group; (d) Blank group and positive control group; (e) Model group and positive control group; (f) Changyu Daotan Decoction group and positive control group. A stands for blank group; B represents model group, C represents Changyu Daotan Decoction group, and C represents positive control group.

**Figure 6:** OPLS-DA replacement trial. (a) Blank and model groups; (b) Blank group and Changyu Daotan Decoction group; (c) Model group and Changyu Daotan Decoction group; (d) Blank group and positive control group; (e) Model group and positive control group; (f) Changyu Daotan Decoction group and positive control group.

**Figure 7:** Cluster analysis. (a) Heat maps; (b) Tree diagram. A stands for the blank group; B represents model group, C represents Changyu Daotan Decoction, and D represents positive control group.

**Figure 8:** *Z*-score. (a) Blank and model groups; (b) Blank group and Changyu Daotan Decoction group; (c) Model group and Changyu Daotan Decoction group; (d) Blank group and positive control group; (e) Model group and positive control group; (f) Changyu Daotan Decoction group and positive control group. A stands for the blank group; B represents model group, C represents Changyu Daotan Decoction group, and C represents positive control group.

**Figure 9:** Correlation heatmap. (a) Blank and model groups; (b) Blank group and Changyu Daotan Decoction group; (c) Model group and Changyu Daotan Decoction group; (d) Blank group and positive control group; (e) Model group and positive control group; (f) Changyu Daotan Decoction group and positive control group.

**Figure 10:** Analysis on metabolic pathways. Based on the KEGG database, the possible upstream and downstream metabolic relationships of the detected substances are drawn on a map.

## Data Availability

The data used to support the findings of this study are included within the article.
